The article "Efficacy and Safety of Stem Cell Combination Therapy for Osteonecrosis of the Femoral Head: A Systematic Review and Meta-Analysis" was published in 2021. Journal: J Healthc Eng.

# Efficacy and Safety of Stem Cell Combination Therapy for Osteonecrosis of the Femoral Head: A Systematic Review and Meta-Analysis

**DOI:** 10.1155/2021/9313201

**Published:** 2021-09-24

**Authors:** Junqiao Li, Peng Su, Jian Li, Gang Chen, Yan Xiong

**Affiliations:** Department of Orthopaedic Surgery, Orthopedic Research Institute, West China Hospital, Sichuan University, 37 Guoxue Lane, Wuhou District, Chengdu, China

## Abstract

**Background:**

The treatment results of core decompression (CD) and biomechanical support are not always satisfactory in osteonecrosis of the femoral head (ONFH). Stem cell therapy has been incorporated into traditional treatment in order to promote bone regeneration. The efficacy and safety of stem cell therapy combined with CD or biomechanical support on advanced and long-term patients with ONFH were unknown. The aim of this study was to assess whether stem cell combination therapy is superior to single CD or porous tantalum rod implantation treatment in ONFH.

**Methods:**

A systematic search of the literature was performed to evaluate all included randomized controlled trials (RCTs) on stem cell combination therapy for patients with ONFH in PubMed, Cochrane Library, Web of Science, and Embase sites. We assessed the quality and risk of bias for the included studies. And the outcomes of Harris hip score (HHS), visual analogue scale (VAS), and adverse events were statistically analyzed.

**Results:**

We included 10 randomized controlled trials, containing a total of 498 patients with 719 hips. Stem cell therapy combined with CD versus CD alone for HHS of ONFH was different (MD = 8.87, 95% CI = [5.53, 12.22], *P* < 0.00001). The combination of stem cell therapy and CD can effectively improve HHS. Similarly, the VAS of the stem cell combination therapy group also differed compared with the control group (MD = −14.07, 95% CI = [−18.32, −9.82], *P* < 0.00001). The result showed that stem cell combination therapy can relieve the pain of patients with ONFH. There was no significant difference in adverse response outcome events between the combination therapy group and the control group (RR = 1.57, 95% CI = [0.62, 3.97], *P* = 0.34).

**Conclusions:**

Stem cell therapy combined with core decompression is an effective and feasible method with few complications in the clinical treatment of early-stage ONFH. Even in the combination of porous tantalum rod implantation and peripheral blood stem cells, stem cell combination therapy is superior to single biomechanical support treatment. But high-quality, large-sample, multicenter, and long-term follow-up RCTs are still needed to corroborate the efficacy and safety of stem cell combination therapy in ONFH treatment.

## 1. Introduction

Osteonecrosis of the femoral head (ONFH) is a prevalent disease in relatively young patients, usually caused by hip trauma, alcoholism and long-term administration of steroid, which may lead to significant hip pain, articular surface collapse, and eventual osteoarthritis [1]. In clinical treatment, various methods are employed to avert or impede the progression of ONFH. The most common form of therapy is core decompression (CD) that has been universally administered for more than 30 years [2]. However, the treatment results of CD are not always satisfactory. This method of reconstructing necrotic areas may result in not only inadequate creeping substitution and but also bone remodeling [3]. Therefore, in order to promote bone regeneration, stem cell therapy has been incorporated into traditional CD treatment. When compared with treating ONFH with CD alone, the combined application of stem cell therapy and CD, in early treatment, has superior analgesic and clinical effects, and can more effectively delay the progress of femoral head collapse [4]. However, the efficacy and safety of these methods have been controversial and have yet to be proven in patients with advanced and long-term ONFH [5, 6].

To investigate the efficacy and safety of stem cell therapy combined with CD or porous tantalum rod implantation in ONFH patients, especially those with advanced stage and long-term follow-up [7], our research systematically retrieved the latest randomized controlled trials on stem cell combination therapy for ONFH according to the PRISMA guidelines [8]. Furthermore, the positive role and improvement of the new technologies in treatment were discussed, with a view of providing clinicians with scientific evidence for the treatment of ONFH patients.

## 2. Materials and Methods

### 2.1. Search Strategy

Two researchers independently searched databases from Cochrane Library, Web of Science, PubMed, and Embase. We integrated published randomized controlled studies of cell therapy for femur head necrosis in any language. The search period was from the date of the database establishment to January 2020. A manual supplementary search was performed before submission. The search terms were adjusted according to each database.

Taking PubMed database as an example, the search terms were as follows: ((Femur^*∗*^ Head Necros^*∗*^ [Title/Abstract]) OR (Necros^*∗*^ of Femur^*∗*^ Head [Title/Abstract]) OR (“Femur Head Necrosis” [Mesh])) AND ((“Cell-and Tissue-Based Therapy” [Mesh]) OR (Cell-[Title/Abstract] AND Tissue-Based Therapy [Title/Abstract]) OR (cell therapy [Title/Abstract]) OR (Cell [Title/Abstract] AND Tissue Based Therapy [Title/Abstract]) OR (Cell Transplantation [Title/Abstract])) AND ((randomized controlled trial [Publication Type]) OR (controlled clinical trial [Publication Type]) OR (randomized [Title/Abstract]) OR (placebo [Title/Abstract]) OR (randomly [Title/Abstract]) OR (trial [Title]) OR (“Clinical Trials as Topic” [Mesh: noexp])).

### 2.2. Criteria for Inclusion and Exclusion

In our qualitative and quantitative analysis, only the studies that satisfied the following PICOS criteria were considered: (1) population: patients with stages I to IV of ONFH diagnosed by the Association Research Circulation Osseous classification (ARCO) [9] diagnostic criteria; (2) intervention: cell therapy combined with core decompression or porous tantalum rod implantation; (3) comparator: single core decompression or porous tantalum rod implantation therapy; (4) outcome: HHS, VAS, and adverse events; and (5) study design: randomized controlled trial (RCT).

We excluded studies with the following criteria: (1) republished studies with similar or identical content; (2) dissertation, conference, and review articles; (3) research in animal and basic experimental literature; (4) non-English published research; and (5) nonrandomized controlled trial or other irrelevant studies.

Two researchers followed the criteria for inclusion and exclusion separately. In case of disagreement, a third researcher intervened to resolve it.

### 2.3. Data Extraction

Two reviewers performed data extraction independently. In case of disputes, differences can be resolved through discussion or third parties until consensus was reached. The extracted information contained baseline information and feature information. The baseline information included: title, study ID, publication country, diagnostic criteria and stages, participants, age, sex ratio, intervention/control group, stem cell source, stem cell counts, the number of hips, and follow-up periods. The feature information included outcome indicators (HHS, VAS), adverse events, effect size, and 95% confidence interval.

### 2.4. Quality Assessment

The included studies were independently evaluated by two researchers in accordance with the Cochrane Handbook for Systematic Reviews of Interventions [10]. Cochrane Collaboration Risk of Bias Tool primarily includes selection (taking into account both allocation hiding and random sequence generation), execution (blinding of both subjects and researchers), measurement (research outcomes blind evaluation), and follow-up (outcome data completeness). A total of seven items in six aspects including gender, reporting, and further potential sources of bias were used to assess the bias risk. For each item, a categorization was specified, counting “low-risk bias,” “high-risk bias,” and “unclear,” with this decision being made in accordance with the bias risk assessment criteria.

### 2.5. Statistical Analysis

Continuous variable values were expressed in mean difference (MD), and a 95% confidence interval (CI) was calculated for both. Regarding dichotomous variables, we used the risk ratio (RR) and 95% CI to describe. When *I*^2^ > 50%, heterogeneity was present within the data; hence, a random-effect model was used. When *I*^2^ < 50%, there was no heterogeneity present; hence, a fixed effects model was used. The findings of the meta-analysis were shown by the forest plot. We utilized RevMan 5.3 software for statistical analysis. *P* < 0.05 was used to evaluate statistical significance. If the number of the included studies was greater than ten, we would use a funnel plot to detect publication bias.

## 3. Results

### 3.1. Search Results

After searching various databases and a manual search method, we retrieved a total of 123 articles. Mechanical check and manual deduplication were performed by EndNote X9, 47 duplicate articles were deleted, 59 articles were excluded from our analysis after abstract screening, and 7 articles were omitted following a full-text screening, resulting in 10 randomized controlled trials being included in our qualitative and quantitative analysis [5, 6, 11–18]. The flowchart is shown in Figure 1.

### 3.2. Study Characteristics

The publication dates of the included RCTs ranged from 2011 to 2018 and belonged to two regions in India [14, 15], one in Iran [16], one in Germany [13], three in China [11, 12, 17], two in Belgium [5, 18], and one in France [6]. All the studies used the ARCO stage as the diagnostic criteria. And the disease stage of the included patients with ONFH was mainly seen in the early phase. A total of 498 participants with 719 hips were included in this study. The longest average follow-up time was up to 25 years. See Table 1 for details.

### 3.3. Quality Assessment

According to the bias risk assessment method recommended by Cochrane Assistance Network, of the 10 studies included, 6 studies [5, 12, 13, 16–18] described the specific random grouping methods, 2 studies [11, 15] mentioned random grouping but did not detail the specific method, and the remaining 2 studies [6, 14] had a high risk of bias; 4 studies [6, 11, 14, 17] showed the unclear risk of bias for the allocation concealment assessment. As for the blinding of participants and personnel, 4 studies [6, 11, 13, 14] did not report whether double-blind information was used, and one study [17] had a high risk of bias; 4 studies [6, 11, 13, 14] showed the unclear risk of bias for the blinding of outcome assessment. Regarding the incomplete outcome data, one study [13] had an unclear risk of bias, and one study [17] showed a high risk of bias. All studies clearly described the selective reporting and had no other risk bias (Figures 2 and 3).

### 3.4. Meta-Analysis Results of HHS

Harris hip score was recorded in six studies [6, 12–15, 17] involving 572 hips. Stem cell therapy combined with core decompression treatment had higher heterogeneity (Chi^2^ = 34.21, *I*^2^ = 85%, *P* < 0.0001) than core decompression alone, and a random effect model was used. The combination treatment group can effectively improve the Harris hip score (MD = 8.87, 95% CI = [5.53, 12.22]), and the difference was statistically significant (*P* < 0.00001). The forest plot is shown in Figure 4.

### 3.5. Meta-Analysis Results of VAS

Five studies [5, 6, 11, 16, 18] including a total of 397 hips reported visual analogue scales. It was evident that stem cell combination therapy yielded a higher heterogeneity than solely administering core decompression or porous tantalum rod implantation (Chi^2^ = 54.20, *I*^2^ = 93%, *P* < 0.00001), and a random effect model was used. Stem cell combination therapy group can effectively relieve the patients' pain (MD = −14.07, 95% CI = [−18.32, −9.82]), with the difference observed between the two groups being statistically significant (*P* < 0.00001). See the forest plot in Figure 5.

### 3.6. Meta-Analysis Results of Adverse Events

The perioperative adverse events were reported in five studies [5, 12, 13, 17, 18]. Of these studies, three studies [5, 12, 18] reported the adverse response outcome events, including the postoperative pain at the great trochanter and iliac crest, hematoma, fever, nausea, infection, and porous tantalum rod displaced. Two studies [13, 17] reported that no adverse events were observed in both groups during the study period. The analysis showed that there was no significant difference in adverse events between the stem cell combination therapy group and the control group (RR = 1.57, 95% CI = [0.62, 3.97], *P* = 0.34). The forest plot is shown in Figure 6.

### 3.7. Publication Bias

As no more than ten published studies were included, it was not possible to assess publication bias for the time being.

## 4. Discussion

### 4.1. Main Findings

Our findings demonstrate that in early-stage ONFH, stem cell therapy combined with core decompression is far more effective than core decompression alone. And the combination therapy has good safety with few complications. Moreover, even in the combination of porous tantalum rod implantation and peripheral blood stem cells, stem cell combination therapy is superior to single biomechanical support treatment.

### 4.2. Effectiveness of Stem Cell Combination Therapy

Stem cell combination therapy can relieve the symptoms of hip pain, improve patients' HHS, halt disease progression, and result in a reduction in the incidence of total hip replacement for the early-stage ONHF patients. This was confirmed in three independent systematic reviews conducted by Papakostidis et al. [19], Piuzzi et al. [20], and Wang et al. [4], respectively. However, in advanced patients, the evolution of necrosis was not significantly improved by stem cell therapy after core decompression [5]. Furthermore, the results of a network meta-analysis study by Yoon et al. [21] questioned the natural course of ONFH by CD treatment. The findings of this study suggested that the small lesions will not collapse, even without treatment being administered. This conclusion took into account that the extent of the decaying component was the primary factor of the necrotic femoral head fracture's collapse. However, even though the progression of osteonecrosis may result from numerous factors [6], an average follow-up time of 25-year prospective randomized study by Hernigou et al. [6] established that bone marrow cell implantation of necrotic lesions may potentially offer an effective treatment for early femoral head necrosis and impede the evolution of ailment, lessen the incidence of femoral head collapse, and elude the arthroplasty even at long-term follow-up.

### 4.3. Safety of Stem Cell Combination Therapy

The probability of adverse complications was extremely low, especially in the aspects of infection, excessive new bone formation, tumor induction, and local complications on the surviving side [13]. Stem cell therapy was safe for the treatment of ONFH. Even after 3–10 years of follow-up, there were no complications related to malignant tumors, bone overgrowth, core tract fractures, perforation of femoral head, deep vein thrombosis, infection, and so forth [7]. Ma et al. [11] conducted a prospective, double-blinded, randomized, controlled investigation. In order to reduce the failure rate, they improved the technology and used autologous bone grafts obtained by ring drilling with bone marrow buffy coat. Hernigou et al. [6] corroborated these findings and noted that computer navigation had the potential to be safely implemented in a basic procedure for the injection of stem cells. They all improved the overall safety of stem cell therapy and reduced the probability of complications. Additionally, Ciapetti et al. [22] demonstrated that, compared with bone marrow mesenchymal stem cells under normal conditions, the proliferation and colonization capacity of these stem cells were significantly enhanced in a hypoxic environment.

### 4.4. Strengths and Limitations

This systematic review was ultimately included in ten studies. All the studies were RCTs of stem cell combination therapy for ONFH, which would provide us with strong evidence for the efficacy and safety of this method in ONFH treatment. Owing to the small number of included studies, we could not make funnel charts to determine publication bias. The heterogeneity in the outcome indicators was large, which may result from certain differences in the included studies in aspects of stem cell concentration, treatment time, and the quality of the literature, leading to greater heterogeneity in each clinical study, and some outcome indicators were not stable.

The findings of this meta-analysis still had certain limitations: (1) the overall quality of the scope of included literature was not high, the sample size was small, and the short follow-up time in some studies may also lead to potential bias; (2) as no more than ten studies were included, publication bias cannot be assessed; (3) publication in English may result in language or regional bias; and (4) there was some heterogeneity in outcome indicators. High-quality, large-sample, multicenter, and long-term follow-up randomized controlled trials are still warranted to corroborate the differences in the efficacy and safety of stem cell combination therapy in ONFH.

## 5. Conclusion

Stem cell therapy combined with core decompression is an effective and feasible method with few complications in the clinical treatment of early-stage ONFH. Even in the combination of porous tantalum rod implantation and peripheral blood stem cells, stem cell combination therapy is superior to single biomechanical support treatment. But high-quality, large-sample, multicenter, and long-term follow-up RCTs are still needed to corroborate the efficacy and safety of stem cell combination therapy in ONFH treatment.

## Figures and Tables

**Figure 1:** Flowchart of literature searching and screening process.

**Figure 2:** Bias graph risk.

**Figure 3:** Bias summary risk.

**Figure 4:** Forest plot of HHS.

**Figure 5:** Forest plot of VAS.

**Figure 6:** Forest plot of adverse events.

**Table 1:** Baseline characteristics of included RCTs.

Study	Year	Country	Study type	Diagnostic criteria	Disease stage	Patient	Age (years)	Sex ratio (M/F)	Intervention/control	Stem cell source	Stem cell counts	Hips	Follow-up (years)
Gangji [18]	2011	Belgium	RCT	ARCO	I/II	19	42.2 ± 2.6	NA	CD + cell therapy	BMMSCs	92.6 ± 22.4 × 10^7^	13	5

Sen [15]	2012	India	RCT	ARCO	I/II	40	NA	NA	CD + cell therapy	BMMSCs	5.0 × 10^8^	26	2

Zhao [17]	2012	China	RCT	ARCO	I/II	100	32.7 ± 10.5	27 : 23	CD + cell therapy	BMMSCs	2.0 × 10^6^	53	5

Rastogi [14]	2013	India	RCT	ARCO	I/II/III	40	34.67 ± 7.02	5 : 2	CD + cell therapy	BMMSCs	1.1 × 10^8^	30	2

Ma [11]	2014	China	RCT	ARCO	I/II/III	39	35.60 ± 8.05	15 : 6	CD + autologous bone graft with BBC	BMMSCs	3.0 × 10^9^	25	2

Mao [12]	2015	China	RCT	ARCO	I/II/III	55	34.60 ± 11.50	17 : 13	Biomechanical support + cell therapy	PBSCs	2.47 ± 0.5 × 10^9^	48	3

Tabatabaee [16]	2015	Iran	RCT	ARCO	I/II/III	18	31.0 ± 11.4	9 : 5	CD + cell therapy	BMMSCs	5.0 ± 2.0 × 10^8^	14	2

Pepke [13]	2016	Germany	RCT	ARCO	II	24	44.3 ± 3.4	10 : 1	CD + cell therapy	BMMSCs	NA	11	2

Hauzeur [5]	2018	Belgium	RCT	ARCO	III	38	48.0 ± 2.8	14 : 5	CD + cell therapy	BMMSCs	19.45 ± 3.51 × 10^9^	23	2

Hernigou [6]	2018	France	RCT	ARCO	I/II	125	18–54	78 : 47	CD + cell therapy	BMMSCs	9.0 ± 2.5 × 10^4^	125	25

NA = not available; CD = core decompression; BBC = bone marrow buffy coat; BMMSCs = bone marrow mesenchymal stem cells; PBSCs = peripheral blood stem cells.

## Data Availability

All data included in this study are available upon request by contact with the corresponding author.
